The article "Imaging features of fibrolamellar hepatocellular carcinoma in gadoxetic acid-enhanced MRI" was published in 2018. Journal: Cancer Imaging.

# Imaging features of fibrolamellar hepatocellular carcinoma in gadoxetic acid-enhanced MRI

**DOI:** 10.1186/s40644-018-0143-y

**Published:** 2018-03-01

**Authors:** Viktoria Palm, Ruofan Sheng, Philipp Mayer, Karl-Heinz Weiss, Christoph Springfeld, Arianeb Mehrabi, Thomas Longerich, Anne Katrin Berger, Hans-Ulrich Kauczor, Tim Frederik Weber

**Affiliations:** 1 Department of Diagnostic and Interventional Radiology, Heidelberg University Hospital, INF 110, 69120 Heidelberg, Germany; 2 Department of Radiology, Zhongshan Hospital, Fudan University, 180 Fenglin Road, Shanghai, 200032 China; 3 Liver Cancer Center Heidelberg, Heidelberg University Hospital, INF 224, 69120 Heidelberg, Germany; 4 Department of Gastroenterology, Infectious Diseases, Intoxication, Heidelberg University Hospital, INF 410, 69120 Heidelberg, Germany; 5 Department of Medical Oncology, National Center for Tumor Diseases (NCT), Heidelberg University Hospital, INF 460, 69120 Heidelberg, Germany; 6 Department of General, Visceral and Transplantation Surgery, Heidelberg University Hospital, INF 110, 69120 Heidelberg, Germany; 7 Division Translational Gastrointestinal Pathology, Institute of Pathology, Heidelberg University Hospital, INF 224, 69120 Heidelberg, Germany

**Keywords:** Diagnostic imaging, Magnetic resonance imaging, Liver neoplasms, Contrast media, Delayed diagnosis

## Abstract

**Background:**

Fibrolamellar hepatocellular carcinoma (FLC) is a rare malignancy occurring in young patients without cirrhosis. Objectives of our study were to analyze contrast material uptake in hepatobiliary phase imaging (HBP) in gadoxetic acid-enhanced liver MRI in patients with FLC and to characterize imaging features in sequence techniques other than HBP.

**Methods:**

In this retrospective study on histology-proven FLC, contrast material uptake in HBP was quantitatively assessed by calculating the corrected FLC enhancement index (CEI) using mean signal intensities of FLC and lumbar muscle on pre-contrast imaging and HBP, respectively. Moreover, enhancement patterns in dynamic contrast-enhanced MRI and relative signal intensities compared with background liver parenchyma were determined by two radiologists in consensus for HBP, diffusion-weighted imaging using high b-values (DWI), and T2 and T1 weighted pre-contrast imaging.

**Results:**

In 6 of 13 patients with FLC gadoxetic acid-enhanced liver MRI was available. The CEI suggested presence of HBP contrast material uptake in all FLCs. A mean CEI of 1.35 indicated FLC signal increase of 35% in HBP compared with pre-contrast imaging. All FLCs were hypointense in HBP compared with background liver parenchyma. Three of 6 FLCs had arterial hyperenhancement and venous wash-out. In DWI and T2 weighted imaging, 5 of 6 FLCs were hyperintense. In T1 weighted imaging, 5 of 6 FLCs were hypointense.

The article "Imaging features of fibrolamellar hepatocellular carcinoma in gadoxetic acid-enhanced MRI" was published in 2018. Journal: Cancer Imaging.

**Conclusion:**

Hepatobiliary uptake of gadoxetic acid was quantitatively measurable in all FLCs investigated in our study. The observation of hypointensity of FLCs in HBP compared with background liver parenchyma emphasizes the role of gadoxetic acid-enhanced liver MRI for non-invasive diagnosis of FLC and its importance in the diagnostic work-up of indeterminate liver lesions.

## Background

Fibrolamellar hepatocellular carcinoma (FLC) is a very rare form of primary hepatic cancer accounting for approximately 5% of all hepatocellular carcinomas (HCCs) [1]. FLCs are composed of well-differentiated neoplastic hepatocytes surrounded by fibrous bands often arranged in lamellar distribution [2]. The molecular basis for the difference between conventional HCC and FLC has recently been elucidated: a translocation resulting in a fusion transcript of the DNAJB1- and PRKACA-genes can be found in all patients with FLC, but not in other forms of liver cancer [3, 4]. Aside from these specific histologic and molecular properties, FLC has decisive clinical features that differ from conventional HCC: FLC develops preferably de novo in the non-cirrhotic liver of young patients without history of chronic liver disease.

From a radiologists’ point of view, it is of utmost importance to distinguish FLC from focal nodular hyperplasia (FNH). FNH is a hepatic tumor that is observed in young patients without chronic liver disease as well, but is always benign, has no potential for malignant transformation and requires no specific therapy. Radiologic discrimination between FLC and FNH can be challenging in magnetic resonance imaging (MRI) because FLC and FNH share important imaging features in pre-contrast and post-contrast scans using conventional extracellular gadolinium-based contrast agents [5–7]. Overlapping imaging features include the presence of a central scar and hypervascularity in arterial phase post-contrast scans. Considering MRI after injection of gadoxetic acid as a liver-specific contrast agent eliminated significantly via the biliary system (Primovist or Eovist; Bayer Vital, Leverkusen, Germany), it is well known that FNH typically shows enhancement during hepatobiliary phase imaging due to hepatocellular uptake of contrast material [8]. To our knowledge, there are incomplete data investigating the behavior of FLC on MRI using liver-specific contrast material.

Primary objective of this study was to investigate presence of enhancement of FLC in post-contrast hepatobiliary phase MRI. Secondary objectives of this study were to describe general imaging features of FLC including morphology and distribution, relative signal intensities in conventional sequence techniques other than post-contrast hepatobiliary phase MRI and presence of accompanying findings.

The article "Imaging features of fibrolamellar hepatocellular carcinoma in gadoxetic acid-enhanced MRI" was published in 2018. Journal: Cancer Imaging.

## Methods

### Study design and study population

This analysis was a retrospective single-center exploratory study on patients that have been identified by chart review of prospectively generated institutional research databases. Approval by the local institutional review board was available. Requirements for inclusion were (1) histology-proven FLC, (2) age ≥ 18 years, and (3) availability of gadoxetic acid-enhanced MRI. If patients had undergone local minimally invasive interventions (i.e. transarterial chemoembolisation [TACE]) prior to gadoxetic acid-enhanced MRI, only viable FLC components were considered. Clinical data were reported via an electronic medical record by the attending oncologists and medical staff. Information included time to FLC diagnosis, primary differential diagnoses on prior imaging studies other than gadoxetic acid-enhanced MRI, and clinical evidence of chronic liver disease. Time to FLC diagnosis was defined as the time period between initial evidence of a hepatic mass and histological diagnosis of malignancy.

### Image analysis

The following sequence techniques covering the liver parenchyma were intended to be included: T2-weighted images without fat saturation (T2wi), pre-contrast T1-weighted images with and without fat-saturation (T1wi), high b-value diffusion weighted images (DWI), and hepatic arterial phase (HAP), portal venous phase (PVP), and hepatobiliary phase (HBP) post-contrast T1-weighted images with fat saturation.

A consensus review of all images was performed by two radiologists. For each imaging sequence, the predominant signal intensities and their homogeneity were visually graded as hyperintense, hypointense, or isointense compared with background liver parenchyma. For quantitative assessment of FLC enhancement, the corrected enhancement index (CEI) was determined for each FLC according to an approach published by Watanabe et al. for hepatobiliary phase liver parenchyma enhancement using the following formula [9]:

$$ \mathrm{CEI}=\left(\mathrm{SI}\ \mathrm{liver}\ \mathrm{HBP}/\mathrm{SI}\ \mathrm{muscle}\ \mathrm{HBP}\right)/\left(\mathrm{SI}\ \mathrm{liver}\ \mathrm{PRE}/\mathrm{SI}\ \mathrm{muscle}\ \mathrm{PRE}\right), $$

where “SI liver HBP” is the FLC signal intensity in HBP, “SI muscle HBP” is the lumbar muscle signal intensity in HBP, “SI liver PRE” is the FLC signal intensity in pre-contrast T1wi with fat saturation, and “SI muscle PRE” is the lumbar muscle signal intensity in pre-contrast T1wi with fat saturation. Signal intensities were assessed using region of interest (ROI) analyses. Ellipsoid ROIs were drawn on representative areas of viable FLC and lumbar muscle on the same slice. Liver and muscle ROIs, respectively, were equivalent concerning size and location for both pre-contrast imaging and HBP. Each measurement was performed three times, and the mean signal intensity was used for CEI calculation.

The article "Imaging features of fibrolamellar hepatocellular carcinoma in gadoxetic acid-enhanced MRI" was published in 2018. Journal: Cancer Imaging.

Predominant enhancement patterns from HAP to PV compared with background liver parenchyma were assigned to either APHE/WO pattern (arterial phase hyperenhancement followed by portal venous hypoenhancement), non-APHE/WO pattern.

Accompanying findings including presence of intralesional necrosis or hemorrhage, bile duct dilatation, bile duct tumor thrombosis, and portal vein tumor thrombosis were analyzed. Presence of intralesional necrosis or hemorrhage was only considered evaluable in patients that had no history of TACE.

## Results

### Patients

Of a total of 13 FLC patients, 6 patients were identified meeting our inclusion criteria. Clinical information on these 6 study patients is summarized in Table 1. Median age at FLC diagnosis was 37 years (range 18–65), and 3 patients were female. FLC diagnosis was delayed in 2 patients with time to FLC diagnosis of 10 months and 20 months, respectively. Delayed diagnosis was associated with advanced tumor stage and early death. These patients were primarily diagnosed with probable FNH at initial presentation at an outside institution. One of these 2 patients presented initially in the early days of clinical introduction of gadoxetic acid. 3 patients had history of TACE with the last intervention 3, 8, and 12 months, respectively, prior to gadoxetic acid-enhanced MRI.

**Table 1:** Clinical information

	#1	#2	#3	#4	#5	#6
Age (years)	52	18	65	26	48	18
Sex	M	F	M	M	F	F
Tumor stage (initial)	pT2 pN0 cM0 (UICC II)	cT1 cN1 cM1 (UICC IVB)	cT1 cN0 cM0 (UICC I)	pT2 cN0 cM0 (UICC II)	cT3b cN0 cM0 (UICC IIIB)	pT3b pN1 cM0 (UICC IVA)
Time to diagnosis (months)	1	10	1	1	1	20
TACE prior to gadoxetic acid enhanced MRI	No	Yes	Yes	No	Yes	No
Treatment	Resection	Sorafenib	TACE, Sorafenib	Resection	Sorafenib	Resection
Survival times	PFS ongoing for 24 months	OS 2 months	OS 29 months	PFS ongoing for 46 months	Lost to follow-up	OS 7 months

*TACE* transarterial chemoembolisation, *MRI* magnetic resonance imaging, *PFS* progression free survival, *OS* overall survival

### Imaging

Gadoxetic acid-enhanced MRI was performed between September 2007 and May 2016. All scanners were 1.5 T devices (Siemens Magnetom Avanto or Siemens Magnetom Aera, Siemens Healthineers, Erlangen, Germany). Specific sequence parameters such as relaxation times and echo times differed between individual MRI protocols. General sequence design is summarized as follows: T2wi was half-Fourier acquisition single-shot turbo spin echo imaging in 5 of 6 examinations and turbo spin echo imaging in 1 examination. Slice thicknesses were 6 mm. T1wi without fat saturation was two-dimensional fast low angle shot imaging in all 6 examinations. Slice thicknesses were 6 mm. DWI was echo planar imaging in all 6 examinations. The highest available b-values were 800 s/mm^2^ in 5 examinations, 600 s/mm^2^ in 1 examination. Slice thicknesses were 6 mm. Pre- and post-contrast T1-weighted imaging with fat-saturation was three-dimensional fast low angle shot imaging in all 6 examinations. Slice thicknesses were 3 mm. HBP was acquired with a median delay after HAP of 18:06 min (range, 16:44–20:43 min). Details on contrast material injection were available for 3 patients. In 2 of these, contrast material was injected with a rate of 1 ml/s and in 1 with a rate of 2 ml/s. Contrast material injection was followed by a saline flush. The contrast material volume was weight dependent and was 10 ml at a maximum with 0.025 mmol/ml gadoxetic acid.

The article "Imaging features of fibrolamellar hepatocellular carcinoma in gadoxetic acid-enhanced MRI" was published in 2018. Journal: Cancer Imaging.

### Lesion features

In 5 of 6 patients the FLC was unifocal. In 1 patient FLC was multifocal with disseminated confluent lesions within the whole liver. In this patient, only the predominant part of the lesion was evaluated. Thus, the evaluated FLCs had a median maximum diameter of 10.5 cm (range, 8.8–14.0). Panels of representative images of each FLC are shown in Figs. 1, 2, 3, and 4. Imaging features are summarized in Table 2.

**Fig. 1:** Image panel of patients #1, #2, and #3 displaying representative sections through individual fibrolamellar carcinoma in non-contrast enhanced techniques including T2 weighted imaging (T2wi), T1 weighted imaging (T1wi), and diffusion weighted imaging using high b-values (DWI)

**Fig. 2:** Image panel of patients #4, #5, and #6 displaying representative sections through individual fibrolamellar carcinoma in non-contrast enhanced imaging techniques including T2 weighted imaging (T2wi), T1 weighted imaging (T1wi), and diffusion weighted imaging using high b-values (DWI)

**Fig. 3:** Image panel of patients #1, #2, and #3 displaying representative sections through individual fibrolamellar carcinoma in contrast enhanced imaging techniques including hepatic arterial phase T1 weighted imaging (HAP), portal venous phase T1 weighted imaging (PVP), and hepatobiliary phase T1 weighted imaging (HBP). In patients with history of TACE prior to gadoxetic acid enhanced MRI (#2, #3) areas of non-viable tumor are indicated in the portal venous phase (arrows) and areas of viable tumor are indicated in the hepatic arterial phase (star)

**Fig. 4:** Image panel of patients #1, #2, and #3 displaying representative sections through individual fibrolamellar carcinoma in contrast enhanced imaging techniques including hepatic arterial phase T1 weighted imaging (HAP), portal venous phase T1 weighted imaging (PVP), and hepatobiliary phase T1 weighted imaging (HBP). In patients with history of TACE prior to gadoxetic acid enhanced MRI (#5) areas of non-viable tumor are indicated in the portal venous phase (arrows) and areas of viable tumor are indicated in the hepatic arterial phase (star)

**Table 2:** Predominant imaging features of fibrolamellar carcinomas

	#1	#2	#3	#4	#5	#6
T2wi	hyperintense	hyperintense	isointense	hyperintense	hyperintense	hyperintense
T1wi	hypointense	hypointense	hypointense	hypointense	hypointense	isointense
DWI	hyperintense	hyperintense	isointense	hyperintense	hyperintense	hyperintense
HAP	hypoenhanced	hyperenhanced	hyperenhanced	hyperenhanced	hyperenhanced	hyperenhanced
PVP	hypoenhanced	isoenhanced	hypoenhanced	isoenhanced	hypoenhanced	hypoenhanced
HBP	hypoenhanced	hypoenhanced	hypoenhanced	hypoenhanced	hypoenhanced	hypoenhanced

*T2wi* T2 weighted imaging, *T1wi* T1 pre contrast weighted imaging, *DWI* diffusion weighted imaging with high b-value, *HAP* hepatic arterial phase post contrast T1 weighted imaging, *PVP* portal venous phase post contrast T1 weighted imaging, *HBP* hepatobiliary phase post contrast T1 weighted imaging

In HBP, all FLCs were hypointense compared with background liver parenchyma. The CEI indicated presence of hepatobiliary contrast enhancement in all FLCs (Fig. 5). The mean CEI averaged over all FLCs was 1.35 indicating a FLC SI increase of 35% in HBP compared with pre-contrast T1wi normalized to muscle SI. Mean SI of FLCs and lumbar muscle and the CEI are shown in Table 3. In HAP, 5 FLCs had predominantly arterial hyperenhancement and 1 FLC had arterial hypoenhancement in lesion components considered viable. In PVP, 4 FLC were predominantly hypointense and 2 FLC was predominantly isointense in lesion components considered viable. The enhancement pattern was considered APHE/WO pattern in 3 FLCs.

The article "Imaging features of fibrolamellar hepatocellular carcinoma in gadoxetic acid-enhanced MRI" was published in 2018. Journal: Cancer Imaging.

**Fig. 5:** Assessment of the corrected enhancement index (CEI) in patient #4. **a** shows the pre-contrast scan. **b** shows the hepatobiliary phase. CEI is 1.51 indicating a signal increase of 51% normalized to lumbar muscle signal intensity. FLC, fibrolamellar carcinoma; HBP, hepatobiliary phase; SI, signal intensity

**Table 3:** Signal intensity and signal intensity ratios

	#1	#2	#3	#4	#5	#6
SI liver PRE	146	114	131	84	96	145
SI muscle PRE	145	151	142	104	112	134
SI liver HBP	136	163	198	133	138	174
SI muscle HBP	99	149	158	109	125	141
CEI	1.38	1.45	1.36	1.50	1.30	1.13

*SI* signal intensity, *PRE* pre-contrast T1 weighted imaging, *HBP* hepatobiliary phase post-contrastT1 weighted imaging, *CEI* corrected enhancement index ([SI liver HBP /SI muscle HBP]/[SI liver PRE/SI muscle PRE])

T1wi and T2wi were available in all patients. In T1wi, 5 FLCs were predominantly hypointense, and 1 FLC was predominantly isointense compared to background liver parenchyma. In T2wi, 5 FLCs were predominantly but heterogeneously hyperintense and 1 FLC was predominantly isointense compared to background liver parenchyma.

DWI and apparent diffusion coefficient (ADC) maps were available in all patients. In DWI with high b-value, 5 FLCs were predominantly hyperintense and 1 FLC was predominantly isointense compared to background liver parenchyma. In ADC map, 4 FLCs were predominantly hyperintense and 2 FLCs were predominantly isointense compared to background liver parenchyma.

Intrahepatic bile duct dilatation, bile duct tumor thrombosis, and portal vein thrombosis were present in 3, 1, and 1 patient, respectively. Intralesional necrosis and intralesional hemorrhage were present in 2 and 0 patients, respectively, of those patients without history of TACE.

## Discussion

In the present analysis on gadoxetic acid-enhanced MRI of 6 patients with histology-proven FLC, contrast enhancement during HBP was present in all FLCs according to calculation of the corrected FLC enhancement index. At visual assessment, all FLCs were hypointense compared with background liver parenchyma. Important imaging features identified frequently in other sequence techniques include heterogeneous hyperintensity in T2wi, hyperintensity in DWI using high b-values, arterial phase hyperenhancement followed by venous wash-out after injection of contrast material, and presence of accompanying findings generally associated with malignancy.

FLC is an infrequent form of HCC mainly occurring equally in female and male patients of younger age without underlying liver disease. Only 20% of FLCs are found in cirrhotic livers [1]. Rarity of FLC and communalities of FLC with other liver lesions may be reasons for preference of benign differential diagnoses in conventional imaging studies and for delayed time to FLC diagnosis. In two of our patients, FLCs were mistaken for FNH at initial presentation. Prolonged time to FLC diagnoses was associated with poor outcome in these cases.

Among benign liver lesions that may be erroneously preferred over malignancy in patients without chronic liver disease, FNH is the most important misdiagnosis in cases of FLC. Mistaking FLC for FNH may have disastrous consequences on patient prognosis if tumor progression during the interval to FLC diagnosis leads to worsening of tumor stage and/or impossibility of curative resection. In patients diagnosed with FLC, positive lymph node status, distant metastatic disease and incomplete resection are associated with decreased survival [10, 11].

The article "Imaging features of fibrolamellar hepatocellular carcinoma in gadoxetic acid-enhanced MRI" was published in 2018. Journal: Cancer Imaging.

Both FLC and FNH are predominantly characterized by generally subtle deviations of signal intensities in pre-contrast T1wi and T2wi compared to background liver parenchyma, arterial hyperenhancement, and presence of a central scar. Imaging features that may favor FLC over FNH in MRI are greater heterogeneity of lesion texture of FLC including necrosis and hemorrhage, hypointensity of the central scar of FLC in T2wi, and portal venous hypoenhancement [12]. Calcifications are reported to be present in approximately 50% of FLCs and not in FNH but are depicted insufficiently in MRI [13]. These imaging features are, however, unreliable discriminators: E.g., the signal intensity of the central scar in T2wi has been shown to be variable [14]. We did not specifically analyze the presence of a central scar and its imaging features in this study, because TACE, which has been performed in 3 of our patients, was considered to affect central scar characterization within treated lesion components.

Gadoxetic acid is a liver-specific gadolinium-based contrast agent that was demonstrated to be of great value for HCC detection in the cirrhotic liver and FNH diagnosis in ambiguous liver lesions [15, 16]. FNHs are characterized by strong uptake of gadoxetic acid leading to iso- or hyperintensity in HBP. Conventional HCCs in the cirrhotic liver are typically hypointense in HBP compared to background liver parenchyma. However, approximately 10% of HCCs in the cirrhotic liver are reported to be not hypointense in HBP due to retained expression of the OATP8 receptor internalizing gadoxetic acid into the hepatocyte [17]. In the non-cirrhotic liver, 5 of 27 HCCs were not hypointense in HBP in a study by Kim et al. [18], but it was not reported if FLCs were included. Thus, precise data on signal behavior of FLC in gadoxetic acid-enhanced MRI are scarce.

In one case report of a pediatric FLC patient the tumor was considered to not show uptake of gadoxetic acid in HBP [19]. In a larger cohort of 37 FLCs only one gadoxetic acid-enhanced MRI was performed, and the tumor was uniformly hypointense in HBP compared with background liver parenchyma [14]. Apart from that, there are apparently only exemplary case presentations available in review articles on liver imaging showing hypointensity of FLC in HBP as well [20–22]. Interestingly, in one illustrative FLC case, uptake of gadoxetic acid in HBP with focal intralesional areas of isointensity was shown by Ringe et al. [22]. To our knowledge, quantitative data on uptake of gadoxetic acid of FLCs or conventional HCC in HBP have not been reported so far. Our case series shows that contrast material uptake may be generally measurable even in FLCs that are in total hypointense compared with background liver parenchyma. This suggests that OATP8 expression is reduced but probably generally present in FLCs.

The article "Imaging features of fibrolamellar hepatocellular carcinoma in gadoxetic acid-enhanced MRI" was published in 2018. Journal: Cancer Imaging.

Concerning DWI in FLC, published experience was very limited so far, but diffusion restriction was suggested to be the most salient finding [12]. The FLCs assessed in our study were qualitatively predominantly isointense (*n* = 1) or predominantly hyperintense (*n* = 4) in the ADC map compared to background liver parenchyma. As other groups have shown that the majority of FNHs are mildly hyperintense in DWI when using high b-values and that the ADC values of FNHs have substantial overlap with the ADC value of background liver parenchyma, we suppose that DWI may not be helpful for distinguishing FLC from FNH either [23, 24].

### Limitations

This single-center study is limited by the small case number due to rarity of the tumor. However, to the best of our knowledge, so far no larger series on gadoxetic acid enhanced MRI of FLC has been reported. Moreover, in 3 of 6 patients TACE had been performed prior to acquisition of gadoxetic acid-enhanced MRI. To ensure a reasonably large study cohort, these patients were not excluded from analysis, but only FLC components were analyzed that progressed after TACE to address possible effects of TACE on lesion features. There was technical heterogeneity of MRI protocols, especially concerning DWI. Thus, ADC value calculation was not feasible. We did not carry out a comparative analysis between FLC and FNH. However, imaging features of FNH including DWI and HBP are well known and analysis of these was suggested not to enhance the data significantly.

## Conclusion

A variable extent of hepatobiliary gadoxetic acid uptake is suggested to be generally present in FLCs. However, the observation of hypointensity of active FLC components in HBP of gadoxetic acid-enhanced liver MRI compared with background liver parenchyma underscores the role of gadoxetic acid for non-invasive diagnosis of FLC and its importance in the diagnostic work-up of indeterminate liver lesions including FNH.

## Abbreviations

ADC: Apparent diffusion coefficient
APHE/WO: Arterial phase hyperenhancement followed by portal venous hypoenhancement
CEI: Corrected enhancement index
DWI: Diffusion weighted imaging
FLC: Fibrolamellar hepatocellular carcinoma
FNH: Focal nodular hyperplasia
HAP: Hepatic arterial phase
HBP: Hepatobiliary phase
HCC: Hepatocellular carcinoma
MRI: Magnetic resonance imaging
PVP: Portal venous phase
ROI: Region of interest
SI: Signal intensity
T1wi: T1-weighted imaging
T2wi: T2-weighted imaging
TACE: Transarterial chemoembolisation
